# A *Medicago truncatula* EF-Hand Family Gene, *MtCaMP1*, Is Involved in Drought and Salt Stress Tolerance

**DOI:** 10.1371/journal.pone.0058952

**Published:** 2013-04-08

**Authors:** Tian-Zuo Wang, Jin-Li Zhang, Qiu-Ying Tian, Min-Gui Zhao, Wen-Hao Zhang

**Affiliations:** 1 State Key Laboratory of Vegetation and Environmental Change, Institute of Botany, The Chinese Academy of Sciences, Beijing, P. R. China; 2 Research Network of Global Change Biology, Beijing Institutes of Life Science, The Chinese Academy of Sciences, Beijing, P. R. China; Iowa State University, United States of America

## Abstract

**Background:**

Calcium-binding proteins that contain EF-hand motifs have been reported to play important roles in transduction of signals associated with biotic and abiotic stresses. To functionally characterize gens of EF-hand family in response to abiotic stress, an *MtCaMP1* gene belonging to EF-hand family from legume model plant *Medicago truncatula* was isolated and its function in response to drought and salt stress was investigated by expressing *MtCaMP1* in Arabidopsis.

**Methodology/Principal Findings:**

Transgenic Arabidopsis seedlings expressing *MtCaMP1*exhibited higher survival rate than wild-type seedlings under drought and salt stress, suggesting that expression of *MtCaMP1* confers tolerance of Arabidopsis to drought and salt stress. The transgenic plants accumulated greater amounts of Pro due to up-regulation of *P5CS1* and down-regulation of *ProDH* than wild-type plants under drought stress. There was a less accumulation of Na^+^ in the transgenic plants than in WT plants due to reduced up-regulation of *AtHKT1* and enhanced regulation of *AtNHX1* in the transgenic plants compared to WT plants under salt stress. There was a reduced accumulation of H_2_O_2_ and malondialdehyde in the transgenic plants than in WT plants under both drought and salt stress.

**Conclusions/Significance:**

The expression of *MtCaMP1* in Arabidopsis enhanced tolerance of the transgenic plants to drought and salt stress by effective osmo-regulation due to greater accumulation of Pro and by minimizing toxic Na^+^ accumulation, respectively. The enhanced accumulation of Pro and reduced accumulation of Na^+^ under drought and salt stress would protect plants from water default and Na^+^ toxicity, and alleviate the associated oxidative stress. These findings demonstrate that *MtCaMP1* encodes a stress-responsive EF-hand protein that plays a regulatory role in response of plants to drought and salt stress.

## Introduction

Calcium ion (Ca^2+)^ is a fundamental transducer and regulator in many processes associated with growth and development as well as response to biotic and abiotic stresses in plants. In plant cells, Ca^2+^ is stored in cell walls and several vesicular compartments (vacuole, endoplasmic reticulum and mitochondria). Under resting conditions, the cytosolic free calcium concentration ([Ca^2+^]_Cyt_) is maintained at approx. 100 nM, which is much less than Ca^2+^ concentrations in the “Ca^2+^ stores” [1]. The movement of Ca^2+^ in and out of cells and organelles can be regulated by Ca^2+^ channels and/or pumps [2], [3]. Upon perceiving cues associated with abiotic and biotic stresses, a rapid increase in [Ca^2+^]_Cyt_ will occur by activating Ca^2+^ channels and/or pumps. Signals related to abiotic stress signals including drought, low and high temperatures, salt and oxidative stress often elicit a rapid elevation of [Ca^2+^]_Cyt_ [4]–[6]. The elevated [Ca^2+^]_Cyt_ is recognized by Ca^2+^ sensors, which in turn relay the information to downstream targets, leading to the alteration of gene expression [7]. The Ca^2+^-dependent proteins regulate physiological and metabolic processes, resulting in phenotypic response to stress [5], [8].

Ca^2+^ sensors are Ca^2+^-binding proteins, and most of the Ca^2+^ sensors contain EF-hand motifs which can bind to Ca^2+^ [9], [10]. The major family of Ca^2+^ sensors includes calmodulin (CaM), calcium-dependent protein kinases (CDPK) and calcineurin B-like proteins (CBL) [11], [12]. Several Ca^2+^-binding proteins have been shown to participate in transduction of signals associated with biotic and abiotic stress. CaM is one of the small, conserved Ca^2+^-binding proteins in eukaryotes [13]. For example, GmCaM4 directly interacts with AtMYB2 in *Arabidopsis thaliana*, and expression of *GmCaM4* in Arabidopsis up-regulates *AtMYB2*-regulated genes, including *P5CS1* (Δ^1^-pyrroline-5-carboxylate synthetase 1) that catalyzes Pro biosynthesis, leading to enhanced tolerance to salt stress [14]. AtCML18, a CaM-like protein, can interact with the C-terminus of AtNHX1, a vacuolar Na^+^/H^+^ antiporter [15]. CDPKs comprise a large family of serine/threonine kinases with kinase domains in the N-terminals in plants [16]. *AtCPK21* is responsive to osmotic stress, whose N-terminal EF-hand pair is a calcium-sensing determinant that is involved in abiotic stress signaling [17]. In addition, CDPKs also play an essential role in response of plants to biotic stress. For instance, silencing *NtCDPK2* renders plants less sensitive to Avr9 virus infection [18]. CBL, a Ca^2+^-binding protein, forms a complex network with their target CBL-interacting protein kinases (CIPK) to regulate a wide range of physiological processes [19], [20]. The expression of *AtCBL1* is markedly up-regulated by drought, cold, and wounding, and is involved in mediation of calcium signaling under certain stress conditions [21]. AtCBL4 (SOS3) can interact with AtCIPK24 (SOS2) by forming a SOS3-SOS2 complex, which in turn activates Na^+^/H^+^ exchanger SOS1 in the plasma membrane of Arabidopsis to pump Na^+^ out of cells. Mutations in the *SOS3* gene render plants hypersensitive to NaCl [22], [23]. Expression of a maize calcineurin B-like protein ZmCBL4 in Arabidopsis confers salt tolerance [24]. In addition, cyclic nucleotide-gated channels (CNGC) may participate in the Ca^2+^-dependent signaling cascades [25]. There have been a number of studies on the functional characterization of Ca^2+^-binding proteins in literature so far. However, there have been few studies focusing on the role of Ca^2+^-binding proteins played in response to abiotic stress in legume species in general and legume model plant *Medicago truncatula* in particular.

In the present study, we isolated a drought-responsive, calcium-binding motif-containing protein gene by the method of suppression subtractive hybridization (SSH), designated *MtCaMP1*, from *Medicago truncatula*, a model plant that has been widely used to study functional genomics of legume plants [26]. We further functionally characterized *MtCaMP1* in response to drought and salt stress by generating transgenic Arabidopsis expressing *MtCaMP1*. Our results demonstrate that expression of *MtCaMP1* in Arabidopsis led to an enhanced tolerance to drought and salt stress. We further explored the physiological mechanisms underlying the enhanced tolerance of the transgenic plants to drought and salt stress.

## Materials and Methods

### Plant growth and treatments

Seeds of *Medicago truncatula* Jemalong A17 were soaked in concentrated H_2_SO_4_ solution for approximately 7 min, and then thoroughly rinsed with water. After chilled at 4°C for 2 d, seeds were grown in a pot (diameter 10 cm) filled with vermiculite: peat soil (2∶1) under controlled conditions (26°C day/20°C night, 14-h photoperiod, and 50%relative humidity) as described by Wang et al. [27].

The effect of abiotic stress on the expression of *MtCaMP1* was evaluated by treatments of four-week-old *M. truncatula* seedlings with drought, salt and osmotic stress, respectively. Drought stress was initiated by withholding water supply to seedlings for varying periods after seedlings were fully watered. Shoots from seedlings suffering from drought stress were harvested after withholding water for 4, 6, and 8 d. Shoots of M. *truncatula* seedlings grown under normal watering conditions were harvested and used as a control. Salt and osmotic stresses were achieved by exposing 4-week-old seedlings to 1/2 MS medium supplemented with 200 mM NaCl and 20% PEG6000 for different periods, respectively.

### Identification of *MtCaMP1* gene and plant transformation

To identify gene fragments in response to drought stress, suppression subtractive hybridization (SSH) was used to construct a cDNA library [28]. SSH was carried out using a PCR-Select cDNA Subtraction Kit (Clontech) according to the manufacturer's instruction. A gene fragment was identified from this cDNA library. The full-length sequence of *MtCaMP1* cDNA was obtained by BLASTn search [29].

The ORF of *MtCaMP1* was amplified with the primers 5′- GAC GGA TCC ATG TCA TTC CTT TCC ACT CT -3′ (*Bam*HI site underlined) and 5′- CAG GAG CTC CTA ACA TAA GAG CAA AAC AC -3′ (*Sac*I site underlined). The *Eco*RI/*Bam*HI -digested product was inserted in the downstream of cauliflower mosaic virus 35S (CaMV 35S) promoter of pSN1301 [30]. After pSN1301: *MtCaMP1* was transformed to *Agrobacterium tumefaciens* GV3101 by electroporation, transformation of *Arabidopsis thaliana* (Col-0) was performed using the *Agrobacterium tumefaciens*- mediated floral dip method [31]. Three independent lines of the T3 generation were randomly chosen for further physiological studies.

### Expression and purification of the EF-hand domain of MtCaMP1

To express and purify the EF-hand domain of MtCaMP1 in *Escherichia coli*, the coding region of the EF-hand domain of MtCaMP1 was amplified by PCR using the primer 5′- AGT GGA TCC TTG AGA GGA GAA AGA AG -3′ containing an *Bam*HI site (underlined), and 5′- GTA CTC GAG ATC CCT GTG TTG AAC AC -3′ containing an *Xho*I site (underlined). The PCR products were digested with *Bam*HI/*Xho*I, and ligated to the C-terminal of glutathione S-transferase (GST) in pGEX-4T-1 (GE). The recombinant plasmid was transformed into *E. coil* BL21. Protein expression was induced with 0.5 mM isopropyl thiogalactopyranoside (IPTG) at 30°C. When the optical density at 600 nm of the culture was reached 0.8 IPTG was added. Bacterial cells were harvested after induction for 6 h by centrifuging the culture at 4000 *g* for 10 min. The purification of recombinant protein was carried out by GST Resin (TransGen).

### Ca^2+^-dependent electrophoretic mobility shift assay

Ca^2+^-dependent electrophoretic mobility shift assay (EMSA) was carried out according to the method descrbied by Burgess et al. and Takezawa [32], [33]. CaCl_2_ at 5 mM or ethylene glycol-bis-(β-amino-ethylether) N,N,N',N'-tetra-acetic acid (EGTA) was added into the sample buffer of GST protein and GST-MtCaMP1 recombinant protein. Proteins were analyzed on 10% polyacrylamide gel electrophoresis under non-denaturing conditions, and stained with Coomassie Brilliant Blue R-250.

### RNA isolation, semi-quantitative and real-time quantitative PCR

Total RNA was isolated using RNAiso Plus reagent (TaKaRa) and treated with RNase-free DNase I (Promega). The total RNA was reverse-transcribed into first-strand cDNA with PrimeScript^®^ RT reagent Kit (TaKaRa).

The semi-quantitative PCR was used to determine the expression level of *MtCaMP1* in transgenic plants. The primers for transgenic Arabidopsis were 5′-CTC AGC ATC CCA GAA TCA A-3′ and 5′-CAG TTC GCA GTC CAT CCC T-3′. *AtActin11* (accession No. NM_112046) was used as an internal control and was amplified with the following primers: 5′-TGT TCT TTC CCT CTA CGC T-3′ and 5′-CCT TAC GAT TTC ACG CTC T-3′. Real-time quantitative PCR (RT-qPCR) was performed using ABI Stepone Plus instrument. Gene-specific primers used for RT-qPCR were as follows: for *MtCaMP1* (5′-CTC AGC ATC CCA GAA TCA A-3′ and 5′-CAG TTC GCA GTC CAT CCC T-3′); for *AtP5CS1* (5′-CTC GCT TAG TTA TGA CGC-3′ and 5′-CTC CTT TCC ACC CTT TA-3′); for *AtProDH* (5′-ATC TTA CCG TTT ACC CG-3′ and 5′-TCA CCG AAG CGT CCA TA-3′); for *AtHKT1* (5′-CAT CTG GCT CCT AAT CCC T-3′ and 5′-ACC ATA CTC GTC ACG CTT T-3′); for *AtNHX1* (5′-GGT TGC CCT TAT GAT GCT TA-3′ and 5′-CTC ACG GAT CTC CAC TTG TC-3′); *MtActin* gene (accession No. BT141409) and *AtActin11* were used as internal controls with primers (5′-ACG AGC GTT TCA GAT G-3′ and 5′-ACC TCC GAT CCA GAC A-3′) and (5′-TGT TCT TTC CCT CTA CGC T-3′ and 5′-CCT TAC GAT TTC ACG CTC T-3′). Primers were designed using the Premier 5 software with the principle to avoid false priming and dimmers. Blasting primers in NCBI and sequencing of PCR produces were used to confirm whether the primers were gene-specific. Each reaction contained 10.0 μL of SYBR Green Master Mix reagent (TOYOBO), 0.8 μL cDNA samples, and 1.2 μL of 10 μM gene-specific primers in a final volume of 20 μL. The thermal cycle used was 95°C for 2 min, 40 cycles of 95°C for 30 s, 55°C for 30 s, and 72°C for 30 s. Three biological and three technological repeats were performed in RT-qPCR. The relative expression level was analyzed by the comparative C_T_ method using the Microsoft Excel 2010 as described by Livak and Schmittgen [34].

### Determination of tolerance to drought and salt stress

Arabidopsis seedlings were planted in pots under the same conditions as described for *M. truncatula*. To determine survival rate after treatment with drought and salt stress, 4-week-old Arabidopsis seedlings were exposed to drought and salt stress by withholding water and irrigating with 200 mM NaCl for 14 days, respectively. After the treatments, plants were transferred to normal growth conditions. The survival rate was determined by scoring the seedlings that failed to grow after recovery from treatments with drought or salt stress. Plants were considered to be dead if all leaves were brown and re-growth did not occur after the plants were transferred to the control growth conditions.

To determinate seed germination rate under osmotic and salt stress, sterile seeds were pointed to 1/2 MS plate (0.8% agar) supplemented with either 300 mM mannitol or 200 mM NaCl at 25°C. Plates that were not supplemented with mannitol or NaCl were used as controls. There were 40 seeds in each plate and the seeds were considered to be germinated at the emergence of the plumule and scored. Seed germination was recorded after 72 h of incubation.

### Determination of water loss rate

For measurements of water loss rate, mature leaves from 4-week-old transgenic and wild-type (WT) Arabidopsis plants were weighed immediately. The leaves were then kept on filter paper in an illumination incubator under the conditions of humidity 40% and temperature of 26°C for varying periods (0, 0.5, 1, 2, 3, 4, 5 and 6 h) and weighed again. Water loss rate was determined by measuring the percentage of fresh weight loss relative to the initial plant weights.

### Determination of H_2_O_2_, malondialdehyde (MDA) and proline (Pro) contents

Four-week-old seedlings withheld water or irrigated with 200 mM NaCl for 6 days harvested for determination of H_2_O_2_ and MDA contents. Seedlings grown in normal conditions were as control. Hydrogen peroxide was measured followed the protocols reported in the literature [35]. MDA content in leaves was determined following the protocol described by Kramer et al. [36]. Pro content in leaves of Arabidopsis was determined as described by Bates et al. [37].

### Measurement of Na^+^ and K^+^ concentrations

Four-week-old seedlings of transgenic and WT plants irrigated with 1/2 MS solution containing 200 mM NaCl for 6 days were harvested and dried at 80°C, and digested with the mixture of nitric acid and hydrogen peroxide using microwave system (MARS, CEM). The digested samples were used to determine K^+^ and Na^+^ contents by ICP-AES (Thermo).

### Statistics analyses

All data were analyzed by analysis of variance using the One-way ANOVA method of SPSS17.0 statistics program. Statistical differences are referred to as significant when *P*≤0.05.

## Results

### Isolation and characterization of *MtCaMP1* gene

Based on sequences of gene fragments isolated from drought-stress suppression subtractive hybridization library, a full-length sequence of a cDNA was obtained by BLASTn (accession No. BT053074). This gene had a 939 bp open reading frame encoding a protein of 312 amino acid residues, with a calculated molecular mass of about 35.5 kDa. Sequence comparison revealed that the putative protein is a calcium-binding motif-containing protein, and is highly homologous to other EF-hand family proteins (Fig. 1). Therefore, this gene was designated *MtCaMP1* (Calcium-binding Motif-containing Protein 1) accordingly.

**Figure 1:** Sequence analysis of EF-hand family proteins. The highly conserved EF-hand motifs of *MtCaMP1* and other known EF-hand family proteins were aligned in panel A. Alignments were performed using the ClustalX2.1 software. X, Y, Z, -Y, -X and -Z represent conserved amino acids of Ca^2+^-binding loop. Phylogenetic tree of these proteins was constructed by MEGA 5 in panel B. The corresponding ID of AtCBL4 (SOS3), ZmCBL4, AtCBL1, OsCDPK7, NtCDPK2, AtCPK21, GmCaM4, AtCML18 (CaM15) and At4G32060 are NP_001190377.1, NP_001150076.1, NP_567533.1, BAB16888.1, CAC82998.1, NP_192381.1, NP_001237902.1, NP_186950.1 and NP_194934.1, respectively.

The EF-hand motif is a helix-loop-helix structure that binds to a single Ca^2+^ ion [9]. This loop consists of 12 residues with the pattern X*Y*Z*-Y*-X**-Z. The residues X, Y, Z, -Y, -X and -Z participate in binding to Ca^2+^ ions, and the intervening residues are represented by asterisk (*). As shown in Figure 1A, MtCaMP1 protein contains two EF-hand motifs which confer EF-hand family proteins the ability of binding Ca^2+^. Similar motifs have been found in many reported EF-hand family proteins. Because the presence of Ca^2+^ would reduce negative charges and lead to a change in conformation, we observed that the recombinant protein was migrated more slowly to the positive pole (Fig. 2). This result validates that the MtCaMP1 can bind to Ca^2+^. Phylogenetic trees based on the full-length amino acid sequences of MtCaMP1 proteins were constructed using the MEGA 5 software (Fig. 1B). The phylogenetic trees show that MtCaMP1 protein had the highest similarity with At4G32060 with unknown function. However, no ortholog of *MtCaMP1* was found in Arabidopsis.

**Figure 2:** Ca^2+^-dependent electrophoretic mobility shift assay of glutathione S-transferasefucata (GST) and GST-MtCaMP1 recombinant protein. Purified protein was run on a 10% non-denaturing polyacrylamide gel in the presence of Ca^2+^ or EGTA. CaCl2 at 5 mM or EGTA was added into the sample buffer.

### Expression patterns of *MtCaMP1* gene

A time-dependent increase in *MtCaMP1* transcripts was observed upon onset of withholding water (Fig. 3A). In addition to withholding water, expression of *MtCaMP1* was also up-regulated by treatments with salt (200 mM NaCl) and osmotic stress (20% PEG6000) (Fig. 3B). Transcripts of *MtCaMP1* were detected in roots, stems, leaves, flowers and pods under non-stressed, control conditions, with the expression being greatest in leaves, followed by roots and stems, lowest in pods (Fig. 3C).

**Figure 3:** Expression patterns of *MtCaMP1* in *M. truncatula*. Expression of *MtCaMP1* in response to drought stress for varying periods was analyzed in panel A. Effect of 200 mM NaCl and 20% PEG6000 on expression of *MtCaMP1* was shown in panel B. Expression patterns of *MtCaMP1* in different organs were shown in panel C. Data are means±SE with three biological replicates.

### Expression of *MtCaMP1* gene enhanced tolerance to drought and salt stress

To functionally characterize *MtCaMP1*, *MtCaMP1* was expressed in *Arabidopsis thaliana* (Col-0) under the control of a CaMV 35S promoter. The transgenic lines were confirmed by hygromycin selection, β-glucuronidase (GUS) staining, and RT-qPCR. Compared with the untransformed WT Arabidopsis, the abundance of *MtCaMP1* transcript was much higher in the transgenic lines (Fig. 4). Three independent transgenic lines (Line 1, 4 and 5) were used for further physiological studies throughout this paper.

**Figure 4:** Analysis of *MtCaMP1* expression level in wild-type and transgenic plants. Expression level of *MtCaMP1* in wild-type (WT) and transgenic plants (line1–5) was monitored by RT-PCR.

Given that the expression of *MtCaMP1* was induced by drought and salt stress in *M*. *truncatula*, we investigated the role of *MtCaMP1* played in response to drought and salt stress by comparing the performance of transgenic plants expressing *MtCaMP1* with WT seedlings suffering from drought and salt stress. After Arabidopsis seedlings of 4-week-old of both transgenic plants expressing *MtCaMP1* and WT were withheld water for 14 d, transgenic plants exhibited higher survival rate than WT (Fig. 5A, B). In addition, the ability of water retention has been widely used as an indicator for drought tolerance in plants [38]. We found that transgenic plants exhibited lower water loss rate than WT (Fig. 5C), indicating that the expression of *MtCaMP1* in Arabidopsis confers the transgenic plants more tolerant to drought stress than WT plants. A similar enhanced tolerance of transgenic plants to salt stress relative to WT plants was also observed (Fig. 6).

**Figure 5:** Effect of drought stress on wild-type and transgenic plants. Phenotypes of wild-type and transgenic plants after withholding water for 14 days were shown in panel A. Survival rates were scored after recovery of watering for 7 days (panel B). Water loss rates were determined at 0, 0.5, 1, 2, 3, 4, 5 and 6 h after drought treatment (panel C). Data are mean±SE with three replicates. Asterisks represent statistically significant differences between wild-type and transgenic lines. * *P*≤0.05, ** *P*≤0.01.

**Figure 6:** Effect of salt stress on wild-type and transgenic plants. Phenotypes of wild-type and transgenic plants after treatment with NaCl for 14 days were shown in panel A. Survival rates were counted after recovery of watering for 7 days (panel B). Data are mean±SE with three replicates. Asterisks represent statistically significant differences between wild-type and transgenic lines. * *P*≤0.05, ** *P*≤0.01.

### Transgenic plants accumulated less H_2_O_2_ and malondialdehyde (MDA)

Plants suffering from abiotic stress often exhibit symptoms of oxidative stress due to excessive accumulation of reactive oxygen species (ROS) and MDA [39]. There were significant increases in H_2_O_2_ and MDA contents in both WT and transgenic plants upon exposure to drought and salt stress, and the stress-induced increases in accumulation of H_2_O_2_ and MDA in the three transgenic lines were significantly less than in WT plants under drought stress (Fig. 7A). A similar less increase in MDA content in the transgenic plants than in WT was also observed when treated with salt stress (Fig. 7B), while expression of *MtCaMP1* in Arabidopsis did not affect MDA metabolism under non-stressed, control conditions (Fig. 7B).

**Figure 7:** Effect of drought and salt stress on contents of H_2_O_2_ and malondialdehyde. H_2_O_2_ contents in wild-type and transgenic plants in control and treatment with drought and salt stress (panel A). Malondialdehyde contents in wild-type and transgenic plants in control and treatment with drought and salt stress (panel B). Four-week-old seedlings withheld water or irrigated with 200 mM NaCl for 6 days were used in the experiments. Data are means ± SE of three biological replicates. Asterisks represent statistically significant differences between wild-type and transgenic lines. * *P*≤0.05, ** *P*≤0.01.

### Transgenic plants accumulated more Pro under drought stress

Accumulation of free Pro is a common phenomenon for plants suffering from abiotic stress such as cold, drought and salt stress [40]. Pro contents in both WT and transgenic plants were comparable under non-stressed, control conditions (Fig. 8A). A marked increase in Pro contents in both WT and transgenic plants was observed upon challenged by drought and salt stress (Fig. 8A). However, the drought stress-induced increase in Pro accumulation in the three transgenic lines was significantly higher than in WT plants (Fig. 8A). In contrast, the increases in Pro contents in WT and transgenic plants were not significantly different under salt stress (Fig. 8A). To further elucidate the mechanism of the drought-induced Pro accumulation, we monitored the changes in transcripts of *P5CS1* and *ProDH* that encode key enzymes responsible for Pro biosynthesis and degradation, respectively. No differences in the abundance of *P5CS1* and *ProDH* transcripts between WT and transgenic plants were found under control conditions (Fig. 8B, C). There were marked increases in *P5CS1* transcripts in both WT and transgenic plants when treated by drought stress (Fig. 8B). However, the drought stress-induced increases in *P5CS1* transcripts in the transgenic plants were significantly greater than in WT plants (Fig. 8B). In contrast to *P5CS1*, *ProDH* transcripts in WT and transgenic plants differed in their response to drought stress such that drought stress suppressed expression of *ProDH* in the transgenic plants, while it had no effect on *ProDH* transcripts in WT plants (Fig. 8C). In contrast to drought stress, both Pro contents and the expression levels of genes encoding Pro metabolism did not differ between WT and transgenic plants in the present of NaCl in the incubation solution (Fig. 8), suggesting that Pro is not involved in the enhanced tolerance of the transgenic plants to salt stress. These results suggest that expression of *MtCaMP1* facilitates Pro accumulation by stimulating Pro biosynthesis and suppressing Pro degradation at the transcript level under drought stress.

**Figure 8:** Drought and salt stress-induced changes in Pro contents. Effect of drought and salt stress on contents of Pro was shown in panel A. The expression levels of genes encoding Pro synthetase (*P5CS1*) and dehydrogenase (*ProDH*) under stress were shown in panel B and C, respectively. Data are mean±SE with three replicates. Asterisks represent statistically significant differences between wild-type and transgenic lines. * *P*≤0.05, ** *P*≤0.01.

### Na^+^ content of transgenic plants under salt stress

Na^+^ is toxic to plants when accumulated excessively in the cytosol when exposed to salt stress. To elucidate the physiological mechanisms by which transgenic plants became more tolerant to slat stress than WT plants, the effects of salt stress on Na^+^ and K^+^ concentrations in shoots of WT and the transgenic plants were investigated. There were no differences in both Na^+^ and K^+^ concentrations in WT and the transgenic plants when they were grown in the control medium in the absence of NaCl (Fig. 9A, B). When the transgenic plants and WT were exposed to solution containing 200 mM NaCl, a marked accumulation of Na^+^ in both WT and transgenic plants was observed (Fig. 9A). However, Na^+^ accumulated in the transgenic plants was significantly less than in WT (Fig. 9A). In contrast to Na^+^, accumulation of K^+^ in both WT and the transgenic plants was equally inhibited under salt stress (Fig. 9B). This led to an increase in Na^+^/K^+^ ratio in both WT and the transgenic lines with the increase being less in the transgenic plants than in WT plants (Fig. 9C). Furthermore, the expression of *AtHKT1* and *AtNHX1* that encode Na^+^ transporters responsible for Na^+^ influx into cytosol and into vacuoles were analyzed in the absence and presence of NaCl by RT-qPCR. As shown in Figure 9D, expression of *MtCaMP1* had little effect on *AtHKT1* transcripts under control conditions. Suppression of *AtHKT1* expression by salt stress occurred in both the transgenic and WT plants, but the salt stress-induced down-regulation of *AtHKT1* expression in the transgenic plants was greater than in WT plants (Fig. 9D). Unlike *AtHKT1*, *AtNHX1* transcripts were more abundant in the transgenic plants than in WT plants under control conditions, and salt stress led to significant increases in *AtNHX1* transcripts in both WT and transgenic plants with the increase greater in the transgenic than in WT plants (Fig. 9E).

**Figure 9:** Effect of NaCl on contents of Na^+^ and K^+^, and expression of *AtHKT1* and *AtNHX1*. Contents of Na^+^ and K^+^ in shoots of wild-type and transgenic plants treated with and without NaCl were shown in panel A and B, respectively. Na^+^/K^+^ ratio was shown in panel C. The expression levels of *AtHKT1*and *AtNHX1* were shown in panel D and E, respectively. Four-week-old seedlings irrigated with or without 200 mM NaCl for 6 days were tested in this experiment. Data are mean±SE with three replicates. Asterisks represent statistically significant differences between wild-type and transgenic lines. * *P*≤0.05, ** *P*≤0.01.

## Discussion

EF-hand family proteins are involved in perception and transduction of calcium signals by binding to Ca^2+^ ions [10], [12]. A number of EF-hand family proteins have been reported to participate in transduction of signals associated with biotic and abiotic stress [5]. For instance, *AtCPK10* plays regulatory roles in modulation of ABA- and Ca^2+^-dependent stomatal movements, such that the *cpk10* mutant is more sensitive to drought stress, while the *AtCPK10-*overexpression lines are more tolerant to drought stress than their wild-type counterpart [41]. Furthermore, AtCBL4 has been shown to activate a Na^+^/H^+^ exchanger SOS1 in the plasma membrane of Arabidopsis by targeting AtCIPK24, and mutation of *AtCBL4* leads to hypersensitivity to NaCl [22], [23]. In the present study, we isolated a gene *MtCaMP1* encoding an EF-hand family protein capable of binding to Ca^2+^ from the legume model plant *M. truncatula*, and evaluated the role of *MtCaMP1* in response to drought and salt stress by generating Arabidopsis plants expressing *MtCaMP1*.

One important finding in the present study is that expression of *MtCaMP1* in Arabidopsis conferred the transgenic plants more tolerant to drought and salt stress. We further explored the physiological mechanisms by which the transgenic plants were more tolerant to drought and salt stress than WT plants. Our results revealed that the transgenic plants accumulated greater amounts of Pro, less amounts of H_2_O_2_, MDA and Na^+^ than WT plants under conditions of drought and salt stress. The accumulated Pro may allow the transgenic plants for more effective osmo-regulation, thus conferring them more tolerant to drought stress by minimizing water loss and maximizing water uptake. The observation that transgenic plants had less water loss rate from leaves than WT plants (Fig. 5C) is consistent with this explanation. There have been reports demonstrating that Pro biosynthesis in plants is regulated by EF-hand family proteins in the literature. For instance, GmCaM4 up-regulates the expression of *P5CS1* by interacting with AtMYB2 [14]. In the present study, we found that expression of *MtCaMP1* in Arabidopsis stimulated Pro biosynthesis and suppressed Pro degradation at the transcriptional level (Fig. 8B, C), thus leading to the enhanced accumulation of Pro under drought stress. In addition to osmo-regulation, Pro has also been suggested to function as a molecular chaperone to stabilize the structure of proteins [42]. Moreover, the less amounts of H_2_O_2_ and MDA in the transgenic plants than in WT plants under drought stress (Fig. 7) may be accounted for by the higher Pro content in transgenic plants than in WT since Pro may protect the transgenic plants from oxidative damage by acting as an antioxidant [42], [43]. Therefore, the greater accumulation of Pro regulated possibly by calcium signals in the transgenic plants under drought stress would confer the transgenic plants to tolerate the drought stress by maintaining favorable water potential and suffering less from oxidative damage.

In contrast to drought stress, accumulation of Pro under salt stress did not differ between the transgenic and WT plants (Fig. 8), suggesting that accumulation is unlikely to account for the differential tolerance to salt stress between WT and the transgenic plants. In this context, we found that expression of *MtCaMP1* in Arabidopsis rendered the transgenic plants accumulated less amounts of Na^+^ than WT under salt stress (Fig. 9). Excessive accumulation of toxic Na^+^ in plant cells, particularly in the cytosol, disrupts K^+^ homeostasis, leading to dysfunction of plant cells. One of the common mechanisms for plants to tolerate salt stress is to minimize Na^+^ influx into cytosol and/or maximize Na^+^ influx into vacuoles [39]. Our results showed that expression of *MtCaMP1* in Arabidopsis led to a marked reduction in Na^+^ accumulation, thus maintaining a higher K^+^/Na^+^ ratio than in WT plants under salt stress (Fig. 9A–C). The lower Na^+^/K^+^ ratio is beneficial for plants to maintain physiological processes under salt stress, thus contributing to the enhanced tolerance of the transgenic plants to salt stress. There are several transporters involved in mediation of Na^+^ flux into and out of cytosol in plants, including SOS1 [44], HKT1 [45] and NHX1 [46]. Mutations in the *AtHKT1* gene suppressed *sos3* mutant phenotypes, and analysis of ion contents in the *sos3hkt1* mutant demonstrated that AtHKT1 is involved in mediation of Na^+^ influx into plant cells [45]. In addition to preventing Na^+^ influx into cytosol, sequestration of toxic Na^+^ in the vacuole by NHX in the tonoplast can also contribute to the enhanced tolerance of plants to salt stress by minimizing accumulation of toxic Na^+^ in the cytosol [46]. In this context, there are reports demonstrating that EF-hand family proteins are involved in regulation of Na^+^ transport mediated by HKT and NHX proteins in the literature. For example, AtCBL4 has been suggested to mediate Na^+^ influx into the cytosol and the vacuole by targeting HKT and NHX, respectively [39]. Conversely, it has been reported that Na^+^/H^+^ exchange activity of AtNHX1 is reduced by AtCML18 [15]. In the present study, we found that the expression levels of *AtHKT1* and *AtNHX1* were significantly reduced and enhanced in the *MtCaMP1*-expressing transgenic plants respectively compared to those in WT plants under the condition of salt stress (Fig. 9D, E). Given that EF-hand family proteins can regulate HKT and NHX by calcium, we speculate that the changes in expression levels of *AtHKT1* and *AtNHX1* in the transgenic plants expressing *MtCaMP1* may also occur in a calcium-dependent manner. It is expected that the down-regulation of *AtHKT1* by expressing *MtCaMP1* would minimize AtHKT1-mediated Na^+^ influx into root cells, while the up-regulation of *AtNHX1* in the transgenic plants would facilitate Na^+^ accumulation in the vacuole. These changes in patterns of Na^+^ transporters at the transcriptional level would allow the transgenic plants to accumulate less toxic Na^+^ in the cytosol, thus conferring transgenic plants more tolerance to salt stress. The reduced accumulation of toxic Na^+^ in the transgenic plants may also account for the observed less accumulation of H_2_O_2_ and MDA in the transgenic plants under salt stress.

In conclusion, we demonstrate that expression of *MtCaMP1*, a gene from *M. truncatula* in Arabidopsis conferred the transgenic seedlings tolerant to drought and salt stress. The physiological mechanisms responsible for the enhanced tolerance to drought and salt stress can be accounted for by enhanced accumulation of Pro due to stimulation of Pro biosynthesis and suppression of its degradation as well as inhibition of Na^+^ accumulation by up-regulating *AtNHX1* and down-regulating *AtHKT1*.

## References

[1] Bush DS (1995) Calcium regulation in plant cells and its role in signaling. In: Jones RL, editor. Annual Review of Plant Physiology and Plant Molecular Biology. 95–122.

[2] SandersD, PellouxJ, BrownleeC, HarperJF (2002) Calcium at the crossroads of signaling. Plant Cell 14: S401–S417.1204529110.1105/tpc.002899PMC151269

[3] TutejaN (2007) Mechanisms of high salinity tolerance in plants. Methods Enzymol 428: 419–438.1787543210.1016/S0076-6879(07)28024-3

[4] TakanoM, TakahashiH, SugeH (1997) Calcium requirement for the induction of hydrotropism and enhancement of calcium-induced curvature by water stress in primary roots of pea, *Pisum sativum* L. Plant Cell Physiol. 38: 385–391.

[5] KnightH (2000) Calcium signaling during abiotic stress in plants. Int Rev Cytol 195: 269–324.1060357810.1016/s0074-7696(08)62707-2

[6] LecourieuxD, RanjevaR, PuginA (2006) Calcium in plant defence-signalling pathways. New Phytol 171: 249–269.1686693410.1111/j.1469-8137.2006.01777.x

[7] SandersD, BrownleeC, HarperJF (1999) Communicating with calcium. Plant Cell 11: 691–706.1021378710.1105/tpc.11.4.691PMC144209

[8] TutejaN, MahajanS (2007) Calcium signaling network in plants: an overview. Plant Signal Behav 2: 79–85.1951697210.4161/psb.2.2.4176PMC2633903

[9] KretsingerRH, NockoldsCE (1973) Carp muscle calcium-binding protein. II. Structure determination and general description. J Biol Chem 248: 3313–3326.4700463

[10] GrabarekZ (2006) Structural basis for diversity of the EF-hand calcium-binding proteins. J Mol Biol 359: 509–525.1667820410.1016/j.jmb.2006.03.066

[11] PoovaiahBW, ReddyAS (1993) Calcium and signal transduction in plants. CRC Crit Rev Plant Sci 12: 185–211.1154006510.1080/07352689309701901

[12] DayIS, ReddyVS, Shad AliG, ReddyAS (2002) Analysis of EF-hand-containing proteins in Arabidopsis. Genome Biol 3: Research0056.1237214410.1186/gb-2002-3-10-research0056PMC134623

[13] YangT, PoovaiahBW (2003) Calcium/calmodulin-mediated signal network in plants. Trends Plant Sci 8: 505–512.1455704810.1016/j.tplants.2003.09.004

[14] YooJH, ParkCY, KimJC, HeoWD, CheongMS, et al (2005) Direct interaction of a divergent CaM isoform and the transcription factor, MYB2, enhances salt tolerance in arabidopsis. J Biol Chem 280: 3697–3706.1556968210.1074/jbc.M408237200

[15] YamaguchiT, AharonGS, SottosantoJB, BlumwaldE (2005) Vacuolar Na^+^/H^+^ antiporter cation selectivity is regulated by calmodulin from within the vacuole in a Ca^2+^- and pH-dependent manner. Proc Natl Acad Sci U S A 102: 16107–16112.1624934110.1073/pnas.0504437102PMC1276053

[16] ChengSH, WillmannMR, ChenHC, SheenJ (2002) Calcium signaling through protein kinases. The Arabidopsis calcium-dependent protein kinase gene family. Plant Physiol 129: 469–485.1206809410.1104/pp.005645PMC1540234

[17] FranzS, EhlertB, LieseA, KurthJ, CazaleAC, et al (2011) Calcium-dependent protein kinase CPK21 functions in abiotic stress response in *Arabidopsis thaliana* . Mol Plant 4: 83–96.2097808610.1093/mp/ssq064

[18] RomeisT, LudwigAA, MartinR, JonesJD (2001) Calcium-dependent protein kinases play an essential role in a plant defence response. EMBO J 20: 5556–5567.1159799910.1093/emboj/20.20.5556PMC125278

[19] KolukisaogluU, WeinlS, BlazevicD, BatisticO, KudlaJ (2004) Calcium sensors and their interacting protein kinases: Genomics of the Arabidopsis and rice CBL-CIPK signaling networks. Plant Physiol 134: 43–58.1473006410.1104/pp.103.033068PMC316286

[20] LuanS (2009) The CBL-CIPK network in plant calcium signaling. Trend Plant Sci 14: 37–42.10.1016/j.tplants.2008.10.00519054707

[21] KudlaJ, XuQ, HarterK, GruissemW, LuanS (1999) Genes for calcineurin B-like proteins in Arabidopsis are differentially regulated by stress signals. Proc Natl Acad Sci U S A 96: 4718–4723.1020032810.1073/pnas.96.8.4718PMC16398

[22] LiuJ, ZhuJK (1998) A calcium sensor homolog required for plant salt tolerance. Science 280: 1943–1945.963239410.1126/science.280.5371.1943

[23] QiuQS, GuoY, DietrichMA, SchumakerKS, ZhuJK (2002) Regulation of SOS1, a plasma membrane Na^+^/H^+^ exchanger in Arabidopsis thaliana, by SOS2 and SOS3. Proc Natl Acad Sci U S A 99: 8436–8441.1203488210.1073/pnas.122224699PMC123085

[24] WangM, GuD, LiuT, WangZ, GuoX, et al (2007) Overexpression of a putative maize calcineurin B-like protein in Arabidopsis confers salt tolerance. Plant Mol Biol 65: 733–746.1788251210.1007/s11103-007-9238-8

[25] TalkeIN, BlaudezD, MaathuisFJ, SandersD (2003) CNGCs: prime targets of plant cyclic nucleotide signalling? Trends Plant Sci 8: 286–293.1281866310.1016/S1360-1385(03)00099-2

[26] CookDR (1999) *Medicago truncatula*-a model in the making! Curr Opin Plant Biol. 2: 301–304.10.1016/s1369-5266(99)80053-310459004

[27] WangTZ, ChenL, ZhaoMG, TianQY, ZhangWH (2011) Identification of drought-responsive microRNAs in *Medicago truncatula* by genome-wide high-throughput sequencing. BMC Genomics 12: 367.2176249810.1186/1471-2164-12-367PMC3160423

[28] WangTZ, ZhaoMG, ZhangWH (2012) Construction and analyses of two suppression subtractive hybridization libraries of *Medicago falcata* and *Medicago truncatula* under drought stress. Acta Prata Sin 21: 175–181.

[29] AltschulSF, GishW, MillerW, MyersEW, LipmanDJ (1990) Basic local alignment search tool. J Mol Biol 215: 403–410.223171210.1016/S0022-2836(05)80360-2

[30] LiCJ, LiangY, ChenCB, LiJH, XuYY, et al (2006) Cloning and expression analysis of TSK1, a wheat SKP1 homologue, and functional comparison with Arabidopsis ASK1 in male meiosis and auxin signalling. Funct Plant Biol 33: 381–390.10.1071/FP0602632689244

[31] ZhangX, HenriquesR, LinSS, NiuQW, ChuaNH (2006) Agrobacterium-mediated transformation of *Arabidopsis thaliana* using the floral dip method. Nat Protoc 1: 641–646.1740629210.1038/nprot.2006.97

[32] BurgessWH, JemioloDK, KretsingerRH (1980) Interaction of calcium and calmodulin in the presence of sodium dodecyl sulfate. BBA-Protein Structure 623: 257–270.10.1016/0005-2795(80)90254-87397213

[33] TakezawaD (2000) A rapid induction by elicitors of the mRNA encoding CCD-1, a 14 kDa Ca^2+^ -binding protein in wheat cultured cells. Plant Mol Biol 42: 807–817.1089052910.1023/a:1006431724090

[34] LivakKJ, SchmittgenTD (2001) Analysis of relative gene expression data using real-time quantitative PCR and the 2^−ΔΔCt^ method. Methods 25: 402–408.1184660910.1006/meth.2001.1262

[35] AlexievaV, SergievI, MapelliS, KaranovE (2001) The effect of drought and ultraviolet radiation on growth and stress markers in pea and wheat. Plant Cell Environ 24: 1337–1344.

[36] KramerGF, NormanHA, KrizekDT, MireckiRM (1991) Influence of UV-B radiation on polyamines, lipid peroxidation and membrane lipids in cucumber. Phytochemistry 30: 2101–2108.

[37] BatesLS, WaldrenRP, TeareID (1973) Rapid determination of free proline for water-stress studies. Plant Soil 39: 205–207.

[38] DhandaSS, SethiGS (1998) Inheritance of excised-leaf water loss and relative water content in bread wheat (*Triticum aestivum*). Euphytica 104: 39–47.

[39] ZhuJK (2002) Salt and drought stress signal transduction in plants. Annu Rev Plant Biol 53: 247–273.1222197510.1146/annurev.arplant.53.091401.143329PMC3128348

[40] AshrafM, FooladMR (2007) Roles of glycine betaine and proline in improving plant abiotic stress resistance. Environ Exp Bot 59: 206–216.

[41] ZouJJ, WeiFJ, WangC, WuJJ, RatnasekeraD, et al (2010) Arabidopsis calcium-dependent protein kinase CPK10 functions in abscisic acid- and Ca^2+^-mediated stomatal regulation in response to drought stress. Plant Physiol 154: 1232–1243.2080532810.1104/pp.110.157545PMC2971602

[42] SzekelyG, AbrahamE, CseploA, RigoG, ZsigmondL, et al (2008) Duplicated *P5CS* genes of Arabidopsis play distinct roles in stress regulation and developmental control of proline biosynthesis. Plant J 53: 11–28.1797104210.1111/j.1365-313X.2007.03318.x

[43] HongZ, LakkineniK, ZhangZ, VermaDP (2000) Removal of feedback inhibition of Δ^1^-pyrroline-5-carboxylate synthetase results in increased proline accumulation and protection of plants from osmotic stress. Plant Physiol 122: 1129–1136.1075950810.1104/pp.122.4.1129PMC58947

[44] ShiH, IshitaniM, KimC, ZhuJK (2000) The *Arabidopsis thaliana* salt tolerance gene *SOS1* encodes a putative Na^+^/H^+^ antiporter. Proc Natl Acad Sci U S A 97: 6896–6901.1082392310.1073/pnas.120170197PMC18772

[45] RusA, YokoiS, SharkhuuA, ReddyM, LeeBH, et al (2001) AtHKT1 is a salt tolerance determinant that controls Na^+^ entry into plant roots. Proc Natl Acad Sci U S A 98: 14150–14155.1169866610.1073/pnas.241501798PMC61183

[46] YokoiS, QuinteroFJ, CuberoB, RuizMT, BressanRA, et al (2002) Differential expression and function of *Arabidopsis thaliana* NHX Na^+^/H^+^ antiporters in the salt stress response. Plant J 30: 529–539.1204762810.1046/j.1365-313x.2002.01309.x

